This article has been retracted.

# The Influence of Cultural Communication on the Psychological Health of University Students in the Environment of Big Data

**DOI:** 10.1155/2022/3037205

**Published:** 2022-10-11

**Authors:** Liu Yang, Jun Liu

**Affiliations:** ^1^Institute of Marxism, Guangxi Arts Institute, Nanning Guangxi 530022, China; ^2^Design Institute, Guangxi Arts Institute, Nanning Guangxi 530022, China

## Abstract

With the progress of information technology and Internet technology, many new media communication technologies are also progressing, and university students are at the forefront of the development of the Internet and the application of cultural communication. Therefore, the impact of modern cultural communication on college students is the most obvious. Time culture communication relies on time communication media, which affects university students' psychological cognition, experience, and mental health level. University students are the high-risk group of mental health problems. At present, most college students are mentally healthy. However, a considerable number of students' mental health is not optimistic. Therefore, paying attention to the impact of culture on college students' mental health plays an important role in the healthy growth of college students. However, a considerable number of students' psychological health is not optimistic. Therefore, paying attention to the impact of culture on university students' psychological health plays an important role in the healthy growth of university students. In this article, 300 university students were randomly selected as the subjects of this study. SCL-90 test and related factors were used to investigate, covering 9 factors. Five common classification algorithms were trained with training sets and evaluated through verification sets. The classifier with the best effect was selected as our algorithm; it is used to discern students with psychological health problems in the test set. The experipsychological results show that precision reaches 0.68, recall reaches 0.56, and F1 measure reaches 0.67. Based on the influencing factors of university students' psychological health, through the analysis of random samples, based on family environment, school environment, community environment, information culture environment, and other factors, this article puts forward strategies to create a warm and progressive family environment, a friendly and positive campus environment, a democratic and scientific community education environment, and a civilized and fair legal environment, so as to properly solve the psychological health problems of university students.

## 1. Introduction

The problem of university students' psychological health has become the focus of attention all over the world, and it is also a major problem faced by all countries in the world. Exploring university students' psychological health teaching model based on big data is helpful to more effectively improve the psychological health level of higher vocational students [1]. In recent years, universities have regularly carried out psychological censuses or assessments, collected basic information of students, and taught psychological courses, which will generate a large amount of diverse data. These fragmented data are inseparable from the factors that affect students' psychological health. The advent of the era of big data has brought unprecedented changes to people's lives, and all walks of life have been impacted to a certain extent. Although “big data” has become a hot word that people are familiar with, it is more concerned by the Internet and the marketing industry [2]. As a cultural industry greatly influenced by big data, the application and value mining of data is still in the initial stage of development. Based on the research on the change of cultural communication of big data, using the research method combining theory and practice, it analyzes the characteristics of cultural communication, the external and internal driving forces of cultural communication reform, etc. and discusses the challenges and challenges brought by big data to cultural communication. Opportunities and strive to put forward to deal with the impact of cultural communication on the psychological health of university students in the context of big data [3].

In this article, the current situation of university students' psychological health and its influencing factors are studied by sampling and collecting the basic information table of students in recent years, SCL-90 data in psychological census and issuing a simple social support questionnaire. Based on the analysis of random samples, this article discusses the family environment, school environment, community environment, information and cultural environment, and other factors and puts forward some targeted strategies, such as creating a warm and progressive family environment, building a friendly and positive campus environment, building a democratic and scientific community education environment, and creating a civilized and just legal environment, to properly solve the psychological health problems of teenagers. At the same time, massive text information from the Internet is introduced to realize transfer learning; data excavation is carried out for data unrelated to the field of psychological health, and TLLR algorithm is used to effectively predict the psychological health status of university students. Therefore, through the analysis of the data in the data set, the attribute values that need to be predicted are found by statistical analysis, and the distribution of attribute values is estimated according to the analysis of similar data [4].

In the era of big data, the channels of cultural communication data are extensive and the cost is low, which makes the data grow exponentially in volume and speed up in transmission by leaps and bounds [5]. Some data of student information can be obtained in the psychological census of university students' enrollment. For a large number of data, how to find useful and decision-making information for students' psychological health education from these data is a very important and complex process. University psychological counseling centers have higher and higher requirements for information processing of computer decision-making and analysis [6]. Facing the increasing expansion of data and the lack of effective means to obtain information, people began to pay attention to data excavation technology. Therefore, we need to be familiar with the development of data excavation and its application in the field of education [7]. The innovation of this article is that

1. The application of data excavation technology to the psychological management system will make effective use of the massive data in students' psychological files, and the decision tree algorithm in data excavation can be used to predict and analyze students' psychological problems; the association rule algorithm can analyze the internal relationship between students' psychological problems and other attributes of students, so that it can provide accurate and useful information for psychological counseling teachers and improve work efficiency
2. This paper applies decision tree excavation technology to the analysis of students' psychological problems, studies data excavation technology based on network environment, especially establishes data excavation server on the Internet, and cooperates with database server to realize the perfect combination of data excavation and mental health education

This article is organized into six sections. The first section is the introduction part, which is based on the influencing factors of university students' psychological health, through the analysis of random samples, and discusses the family environment, school environment, community environment, information and cultural environment and other factors, aiming to solve the problem of university students' psychological health. The second section mainly summarizes the relevant literature, summarizes the advantages and disadvantages, and puts forward the research ideas of this article. The third section introduces in detail the application of university students' psychological health management in the context of big data era and mentions the comparative application of algorithms. The fourth section analyzes the influencing factors of university students' psychological health, especially the sample data set. The fifth section is the optimization strategy of university students' psychological health development. The sixth section is the conclusion, summary, and outlook.

## 2. Related Work

The researchers expounded the concept of big data. Zhang and Jia proposed a new method to obtained students' depression scores through depression questionnaire and established a more accurate prediction model to identify the psychological state of depressed groups [8]. On the other hand, Xia proposed the goals, contents, and strategies of digital campus construction under the background of big data [9]. Xuan observes the significant relationship between emotional expression and the individual characteristics of searchers; the investigation of users' emotions in the search process showed that users with happy emotions invested a lot of time in searching and viewing search solutions [10]. Gao analyzed the employment value orientation of university students based on big data and proposed corresponding guidance strategies [11]. Although the establishment of psychological archives has attracted the attention of many schools, from the current application practice, the quality and quantity are not satisfactory. Researcher Xia conducted a cross-sectional historical meta-analysis on the mental health level of college students in recent 10 years, and the results showed that the overall level of mental health of college students was gradually improving [12]. In terms of gender differences, the trend of improving the psychological health level of boys is higher than that of girls. In the research of influencing factors of psychological health, Ming and Long think that when people are in poverty, the improvement of economic development level can enhance the harmony of psychological health, but when the economic development level reaches a “turning point”, the relationship between psychological health and economic development level will become complicated [13]. In view of the increasing environpsychological uncertainty of the whole society, Chen believes that anxiety has become a basic social psychologicality [14]. Xiaojun and Zheng believe that in today's network society or information society, information has become the direct production object, which leads to uncertainty becoming the essential characteristic of network society [15]. The unprecedented abundance of information on the Internet and the extremely fast speed of communication and diffusion have further strengthened the uncertainty of cultural communication. Haixia and Qing believe that, for university students, the upward mobility demand and the uncertainty of the environment together cause the “class anxiety” of contemporary university students [16]. Shihuan believes that the process of social transformation has brought more environpsychological uncertainty, which is a major reason for the decline of adolescents' psychological health [17]. From the psychological point of view, uncertainty means that individuals cannot make an accurate assessment of the future, so they cannot make preparations in advance, which leads to students' anxiety.

## 3. The Application of University Students' Psychological Health Management under the Background of Big Data Era

### 3.1. Characteristics of Cultural Communication in the Era of Big Data

Compared with traditional media, the era of big data has obvious characteristics of media transformation, which are embodied in the following aspects:

(1) *Thematic*. In the context of big data, the hotspots and sensitive information of cultural communication tend to be blurred. Due to the large amount of information and faster updating, the collection and analysis of data cannot be precise, but the theme is set by ordinary people as the subject of reception. It shows the theme of large capacity, short cycle, and fast production [18].

(2) *Abundance*. Due to the universality, equality, and openness of big data, recipients of different age groups can share personal and group information anytime, anywhere, regardless of their status.

(3) *Reality*. The main body of cultural communication is no longer limited to professional media practitioners but maximizes the freedom to select thematic content and style characteristics and can more freely reflect the reality of life [19]. Spontaneous cultural communication subjects get rid of the dogma of communication theory, form a simple cognition of objective things, get through the convenient channel of big data platform with unique emotional expression, and easily get the communication themes close to life.

(4) *Fissibility*. In cultural communication, with the help of existing social media such as Weibo, WeChat, and QQ, the core supporting role of data analysis technology is brought into play, so as to achieve the communication validity of instantly driving culture to radiate from one social group to another.

(5) *Intelligence*. Big data technology spans the distance between time and space, spreads culture through virtual data magic, and realizes the intelligent synchronization between the virtual world and the real world. Communicators and receivers participate in the release scope and in-depth discussion that is not limited by time and space. Through the push of big data, the whole process from cultural interaction to cultural identity can be completed in the shortest time, and the communication effect can be maximized. The future will be a world that dares to change and innovate constantly, and intelligence will become the trend leading the future communication field [20–24].

### 3.2. Data Mining Algorithm Based on Big Data

In the actual use of the psychological management system, the task of screening students with mental disorders is basically completed by the psychological measurement scale. However, the diagnosis of students with mental disorders cannot be determined only by the score of a single measurement scale, and the scale is only an auxiliary tool. It is our desire to mine and search out regular and meaningful patterns from the database. Therefore, using data excavation technology to analyze and diagnose more scientifically and accurately can really help psychological counselors and counselors do a good job in mental health education and can really help psychological students to solve mental problems as soon as possible.  Figure 1 shows a data excavation model, which represents the basic process of data excavation.

Using the fast, predictable, accurate, and practical application value of big data technology, we can quickly and accurately determine the state and degree of crisis, so as to effectively formulate crisis intervention plans and reduce or eliminate crises. In the process of data excavation, select the appropriate data excavation algorithm to analyze the input data after preprocessing and use the efficient data excavation algorithm to scan the data set repeatedly or once to produce the desired mining results, so as to find the correlation between attribute values and obtain a new cognition that is more realistic than the original cognition.

In order to obtain the ideal mental health evaluation results of college students, a big data-driven mental health evaluation model of college students is designed, which fully considers the big data-driven background, applies the efficient data clustering method to big data, establishes the mental health evaluation index system of college students, determines the weight of each index in the evaluation index system, and uses the fuzzy comprehensive evaluation method to evaluate the mental health of college students, and to realize the quantification of College Students' psychological state and provide effective reference basis for colleges and universities to formulate educational courses and psychological counseling, as shown in Figure 2. Applying the big data-driven data clustering method to the mental health evaluation data of college students, we need to calculate the similarity of different texts in the massive big data and obtain the similarity by counting the number of the same feature words between different texts.

In the psychological management system, a large number of psychological measurement scales are introduced. The data in these scales are added by psychologists from relevant aspects. The items in the scales reflect some symptoms, requiring subjects to make independent self-assessment that is not affected by anyone, so as not to affect the accuracy of analysis. The information collected by establishing psychological archives may not cover all the information needed for the study. In addition, human factors may also lead to the deviation and mutilation of data records. Students' incomplete information will be affected by their unclear understanding of the project and their own evaluation. Therefore, the information obtained by students using a single scale cannot determine the mental health status of students. More scientific and accurate data will be obtained after comprehensive analysis of students' basic information and influencing factors. Therefore, we plan the overall framework of the student mental health problem recognition algorithm based on multisource data, as shown in Figure 3.

In the process of freshmen's psychological survey in recent years, the psychological measurement analysis results show that the proportion of individuals with abnormal psychology is very large, which can not screen out the individuals with real psychological abnormalities and can not well reflect the actual mental health status of students. Most of them are measured by SCL-90 psychological measurement scale and UPI measurement scale. Such results also directly affect the application of data excavation technology. Therefore, the method of linear fitting can be considered to correct the data, so as to improve the measurement results and provide a favorable guarantee for data excavation.

### 3.3. Introduction to Different Algorithms

The most critical technique in the construction of a decision tree is the selection of split attributes. There are often many attributes in the data set. For some high-dimensional data sets, there are even thousands of attributes. How to choose the best attribute is a decision tree. The research focus is, among several attributes, which attribute is preferentially selected for splitting. C4.5 algorithm is the improvement of ID3 algorithm and the basis of more decision tree algorithms. The method of constructing decision tree is top-down recursive construction. Select an attribute in the training set according to a certain strategy, divide the data set into several subsets according to each value of the attribute, and satisfy that all data in each subset have the same attribute value on the selected attribute, and then recursively perform subsequent processing in each subset. The binary decision tree obtained by C4.5 algorithm under this unbalanced data set can fully meet the needs of students' mental health analysis. The calculation of the information entropy is shown in Formula (1).

(1) $$\begin{array}{c} \text{entropy}\left(G\right)=-\overset{m}{\underset{i=1}{\sum }}p_{i}\log_{2}\;p_{i}. \end{array}$$

Among them, *m* represents the number of categories in data set *G*, *p*_*i*_ represents the probability of the *i*-th category, and the smaller the value of *entropy*(*G*), the higher the purity of *G*.

The implementation of the SCL-90 algorithm is based on the completion of supervised learning on labeled training, so the basic model needs to be determined first. The model has a wide range of choices, and the logistic regression model (LR) is selected in this article. Under this model, the classification is done using the discriminant based on the logical distribution. The mathematical definition of the logical distribution is as follows:

(2) $$\begin{array}{c} p\left(y\left|x\right.\right)=\frac{yx^{T}w}{1+yx^{T}w}. \end{array}$$

In corpus |*y*, *x*|, the LR model is

(3) $$\begin{array}{c} w=\arg_{w}\min\overset{n}{\underset{i=1}{\sum }}\log\left(1+\left(-yx^{T}w\right)\right). \end{array}$$

The calculation result of the above formula is a linear function. At the same time, starting from the LR model, its characteristics are independent of each other. However, for text information mining, lexical co-occurrence information is a feature significantly different from general tasks. Therefore, it needs to be enhanced. This article establishes a relationship graph between domain independent features and domain specific features. The adjacency matrix of this graph is

(4) $$\begin{array}{c} A=X^{T}X-\mathrm{diag}\left(X^{T}X\right). \end{array}$$

To solve this problem, this article uses the OWL-QN algorithm. First, the objective function is rewritten in the form of adding the loss function and the L1 norm:

(5) $$\begin{array}{c} f\left(A,B\right)=L\left(a,B\right)+R\left(w\right). \end{array}$$

The loss function of the TR model is

(6) $$\begin{array}{c} L\left(w\right)=\overset{n}{\underset{i=1}{\sum }}\log\left(1+\left(-yx^{T}w\right)\right)+\frac{1}{2}\beta \overset{n}{\underset{i\neq 1}{\sum }}{\left(w-c\right)}^{2}. \end{array}$$

The Pearson coefficient indicates the ratio of the same number of feature words in different texts to the smaller value of the total number of feature words, that is, the text similarity. The clustering index is extended by the self-adaptive method, a fixed threshold is set, and the texts whose text similarity is higher than the threshold are clustered into one class, and the clustering results obtained are used as the evaluation index. The similarity of relevant evaluation indicators is

(7) $$\begin{array}{c} {\text{p}}_{\alpha ,\beta }=\frac{\mathrm{cov}\left(\alpha ,\beta \right)}{\delta_{x,y}}=\frac{E\left(\alpha ,\beta \right)-E\left(\alpha \right)E\left(\beta \right)}{\sqrt{E\left(\alpha^{2}\right)-E\left(\beta^{2}\right)}}, \end{array}$$

where *α*, *β* is the two random variables, cov(*α*, *β*) is the covariance between *α*, *β*, and *δ*_*x*,*y*_ is the standard deviation between *x*, *y*, and *E* is the mathematical expectation in statistics. In order to improve the efficiency of data excavation, it is usually not necessary to use all the data in the system. Some data objects and data attributes have no impact on the establishment of model acquisition mode. Before data excavation, a lot of work needs to be done in the research stage. Data extraction is designed according to the collected information, and the required data sources are determined for the defined project tasks, from which data is collected and extracted, which not only simplifies the data. It can also make the hidden laws and internal connections appear. Therefore, it is necessary to select data effectively.

Since we can calculate the values of *Z*, and values (these two values may be called empirical values) according to the given training sample set, assuming that the measured SCL-90 value of a certain student is *X*, and the UPI result value is *Y*, you can use the formula

(8) $$\begin{array}{c} Z=100-\left(k_{1}X+k_{2}Y\right). \end{array}$$

To obtain the value of students' psychological health *Z* (the meaning of this value is the same as that of the subjective evaluation value), which can be used as the evaluation basis of students' psychological health. After the results are obtained through calculation, the obtained student psychological health status value *Z* should be compared with the system technical indicators to judge whether the current data correction meets the predetermined requirements. Therefore, error analysis is carried out:

The absolute error is

(9) $$\begin{array}{c} \sqrt{\frac{1}{n}\overset{N}{\underset{i=1}{\sum }}e_{i}}=2.398. \end{array}$$

The relative error is

(10) $$\begin{array}{c} \sqrt{\frac{1}{n}\overset{N}{\underset{i=1}{\sum }}{\left(\frac{e_{i}}{b_{i}}\right)}^{2}\times 100\%=19.328\%}, \end{array}$$

where *N* is the total number of samples. After the error analysis, it shows that after the linear correction, the accuracy of the students' psychological measurement can also meet the application requirements.

## 4. Analysis of the Influencing Factors of University Students' Psychological Health

In the SCL-90 survey, it can be seen that there are changes in university students' gender, place of origin, and family economic status, and the somatization index of university students is far lower than the norm, which indicates that the psychological health problems of university students are mainly manifested in their emotions and thinking and have not developed to the point of somatization. Therefore, in the process of daily education, emphasis should be placed on education and prevention to promote the healthy development of university students. For educational institutions such as schools, it is necessary to set up psychological counseling or psychological health departments to regularly guide and intervene the psychological health problems of university students. Then, only by analyzing the influencing factors of students' psychological health can we solve the problem and help university students to correct their psychologicality and maintain a healthy psychological state:

(1) *Family factors*. Most parents have set high learning goals for their children and designed their children's future career direction, placing all the hope of changing the fate of the whole family on their children and continuing to put pressure on them. In such a high-pressure growth environment, many young people are prone to unhealthy psychology, and it is difficult to achieve comprehensive and healthy development.

(2) *School environpsychological factors*. In order to maximize the enrollment rate and employment rate, the school pays more attention to the students' academic scores, thus ignoring the students' psychological guidance education, which further causes different degrees of psychological pressure on the students.

(3) *Social factors*. The current social graduates are overwhelming, the employment situation is severe, and the rise of the service industry and the social and cultural atmosphere created by related industries has adversely affected the psychological health of young people. Many media information has misled university students' cognition.

### 4.1. Analysis of Sample Datasets

In order to better correspond to this proportional relationship, this article uses OMD, HCR, and TGM domain independent text sets to realize transfer learning. Because OMD, HCR, and TGM datasets have more regular data structures and richer vocabulary, the training and testing effects are better. Compared with logistic regression model and naive Bayesian model, their accuracy is improved by 10.19% and 4.11%, respectively. This algorithm realizes the transfer learning from OMD, HCR, and TGM datasets to university students' psychological health datasets. In addition to the accuracy of the analytical model, the article also analyzes two parameters that affect the effect of transfer learning *λ*、*β*. The influence of model performance is simulated, and the results are shown in Figures 4–5.

It can be seen from Figure 4 and Figure 5 that the accuracy of TL algorithm on HCR data set is lower than that of OMD and TGM models, which is due to the fact that the coincidence degree of OMD data is higher than that of HCR model. About *λ* it is insensitive to the accuracy of the model within the value range of [0.7, 0.9]. About *β* it is also insensitive to the accuracy of the model within the value range of [0.3, 1.0]. Therefore, in general, TL is insensitive to the changes of model migration parameters, which greatly reduces the training requirements of the model.

Due to the different qualities of students in various majors, the data in the system has particularity. Here, we take the psychological management system database of our students as an example to carry out a simple data extraction work. In order to facilitate the establishment of the decision tree model, from the many attributes in the student psychological management database of our school, select the attributes that are more relevant to the mining task, while other attributes that are not related to the mining task will increase the time and space of mining calculation to a certain extent. Therefore, the irrelevant attribute values should be removed when mining such data. We analyze the record data of students' mental health status, so as to deduce what factors affect students' mental health status. From the derived rules, psychological counselors can judge which aspects of mental health education and intervention should be strengthened to enable students to improve their ability of self-growth. In this paper, we choose precision, recall, and F1 measure as evaluation indicators, and their application to the model performance comparison is shown in Figure 6 below.

Table 1 lists the experipsychological results of three different feature combinations on deep psy model. In order to facilitate the analysis of the changes of the experipsychological results, we visualize the data in Table 1, as shown in Figure 7. First, the experipsychological result of feature set 1 is the best. Secondly, with the reduction of feature types, the experipsychological effect gradually becomes worse, especially the decline of feature set 4 is large, because the number of consumption features is large, which has a great impact on the experipsychological results. The experipsychological results show that we conclude that many objective factors have an impact on mental health by analyzing and mining information.

### 4.2. Analysis of Psychological Health Factors

In this article, 200 university students were randomly selected as the subjects of this study. SCL-90 test and related factors were used to investigate, covering 9 factors: somatization, obsessive-compulsive symptoms, interpersonal sensitivity, depression, anxiety, hostility, terror, paranoia, and psychosis. Five common classification algorithms were trained with training sets and evaluated through verification sets. The classifier with the best effect was selected as our algorithm. It is used to distinguish students with psychological health problems in the test set. In the process of carrying out the research, this article takes the average score of each factor of SCL − 90 ≥ 3 as the evaluation standard of psychological problems. During the survey, 88 teenagers in the sample have at least one factor exceeding 3 points, so the detection rate is 16.92%. According to statistics, the top five factors include compulsion (3.22%), interpersonal sensitivity (2.80%), depression (1.27%), paranoia (1.06%), and hostility (1.95%), as shown in Figure 8.

In the process of analysis, the closer the tolerance is to 1, the better the result, and the variance inflation factor is less than 10, and the smaller the better. From the final results of the collinearity study, there was no collinearity among the four studied variables, and the final results all showed that the predictors were fully incorporated into the regression equation. At the same time, the constant of SCL-90 is 1.239, and the values of the equation model are 0.349, 0.459, and 0.897, respectively.

## 5. Optimization Strategies for the Development of Psychological Health of University Students

Under the spread of diversified culture, schools and society need to create a more harmonious environment for university students' psychological health, so we need to do the following:

1. Harmonious family environment. In the process of family education, simple preaching should be avoided, and heuristic education should be used to guide their psychological health development on the basis of good communication, so as to create a good family education atmosphere. Parents should consider their children's development comprehensively, provide them with diversified choices, and conform to each child's different development needs
2. A positive and friendly campus environment. While consolidating its own modern educational thought and students' knowledge and culture teaching, the school should pay attention to the education of students' thought and personality, constantly create a campus environment conducive to the improvement of students' own quality, and construct a perfect lifelong education learning thought. Through the diversified quality-oriented education model, we can help university students broaden their horizons, strengthen their sense of mission, and cultivate positive interests in the big classroom of society, so as to improve their own quality and practical ability in rich practice
3. The spread of socialized culture and the improvement of education. From the perspective of data capture and analysis of big data technology, roles, situations. and behaviors are important representations of cultural communication to build a media society. The changes of roles, situations, and behaviors in the media society are intertwined, forming the external power of cultural communication change under the background of big data. From the source and policy, the state and government should strengthen the audit of online games and mobile apps, and add antiaddiction factors

## 6. Conclusions

The influence of cultural dissemination of the times on university students has both good and bad aspects. Those unadvocated parts of the culture of the times will make a huge change in students' attitude towards life. University students are like a piece of “white article” that has not yet entered the world. Their ability to judge right and wrong information is immature, and their ability to resist bad information is also limited. Therefore, poor culture can easily invade students' minds and affect their physical and psychological health. Health has a huge impact. And a good culture of the times is conducive to the formation of correct values for university students, and to live a full university life. Therefore, in the diverse and rich era environment, university students should improve their ability to distinguish good and bad cultures and promote the development of physical and psychological health. Based on the role of big data technology, analyze the influence of factors and provide guidance and reference for the development of university students' psychological health.

## Figures and Tables

**Figure 1:** Model of big data excavation.

**Figure 2:** Structure diagram of mental health crisis prevention system.

**Figure 3:** Algorithm framework of student psychological health problem identification based on multisource data.

**Figure 4:** Relationship between *λ* and classification accuracy.

**Figure 5:** Relationship between *β* and classification accuracy.

**Figure 6:** Comparison of model performance indicators.

**Figure 7:** Comparison of three characteristic data results.

**Figure 8:** Evaluation of the training set of each factor.

**Table 1:** Experipsychological results of three different feature combinations on the deep psy model.

Dataset	Precision	Recall	F1-measure
1	0.68	0.79	0.74
2	0.78	0.8	0.79
3	0.76	0.74	0.7
4	0.65	0.73	0.63

## Data Availability

The figures and tables used to support the findings of this study are included in the article.
